# Fusion Evaluation of College Cultivation by Adaptive Multivariate Neural Network Model

**DOI:** 10.1155/2022/1449753

**Published:** 2022-08-08

**Authors:** Shaoyong Hong, Chun Yang, Shitong Ye, Shaohong Chen

**Affiliations:** ^1^School of Data Science, Guangzhou Huashang College, Guangzhou 511300, China; ^2^School of Accounting, Guangzhou Huashang College, Guangzhou 511300, China; ^3^School of Foreign Languages, Guangzhou Huashang College, Guangzhou 511300, China

## Abstract

The quality of graduates is the key factor in evaluating the cultivation effect of colleges and universities. Quantification of whether the graduates qualify for their working post in companies and industries provides conduction for further college cultivation reform enhancement. In this work, we proposed an adaptive multivariate neural network architecture for fusion evaluation of college student cultivation. Specifically, we designed a questionnaire to collect data on the current working status of 1231 graduates and recorded 32 in-school training items categorized into four different modules. For quantitative evaluation, 10 indices of career-require competence were set to describe the graduates' job abilities. The fused contribution of the in-school training items to the career-required competence was predicted by the multivariate network model with the linking weights adaptively trained. A comprehensive contribution matrix was generated by discrete PCA multivariate transforming to provide a digital reference for the network training. A 7-level scoring system was designed for quantifying the contribution matrix. For model optimization, the network structure was tuned by testing a different number of hidden nodes. The model was trained and optimized to reveal the direct correlation between college cultivation and job-required abilities. Experimental results indicated that the methodology we proposed is feasible to evaluate the cultivation mode in colleges and universities, theoretically and technically providing positive directions for colleges and universities to make their cultivation reforming, as to enhance the quality of their graduates.

## 1. Introduction

With the daily changing informed society, the current competition is reflected in the competition for high-quality talents [1]. Nowadays, millions of students receiving higher education graduate from colleges and universities every year. The graduates would face fierce competition when they are looking for a job [2]. Colleges and universities play a significant role in cultivating their students to high-end information talents. They are tackling the bottleneck issue of improving the students' job career-required competence ability [3, 4]. Thus, it is much important to evaluate how in-school cultivation supports the graduates' career-required competence by investigating machine learning methods and intelligent models [5].

In colleges and universities, some compulsory and elective courses are set up for the students to take part in when they are undergraduates to expand their knowledge concerns and refine their basic knowledge structure [6, 7]. A lot of extracurricular practical activities are available for any student who intends to participate, such that the students can gain practical experience and raise their self-awareness in the activities [8, 9]. The students' personal ability can be trained under the interaction of in-class courses and extracurricular activities. A series of in-school training items are introduced, then the in-school cultivation can be qualified with scorings in these items so as to comprehensively evaluate their job competence [10].

Actually, career-required job competence cannot be directly measured. In statistical concepts, competence can be implicitly explained by some practical factors for employment postevaluation [11]. These factors may refer to many aspects, such as the working location, working post, salary, and promotion times. Based on different factors, the career-required job competence and the in-school training items can be scored.

Adaptive neural network architecture is built upon targeting to score the in-school training items contributing to the indices of career-required competence. The network is comprised of a large number of connected nodes. Each node performs a simple calculation [12]. It excels at handling nonnormally distributed multivariate problems and has led to many recent advances in artificial intelligence [13]. The model is usually designed to deliver the white data feedforward and the error feedback [14]. The optimization criterion in neural networks is to minimize the error on the training or test set [15]. A neural network is widely applied to the fields of image analysis, environmental detection, and medical diagnoses [16–18]. In the application, the network link weights are automatically trained from the input data using a data-driven learning strategy [19].

In the modeling process, the adaptive multivariate network architecture is designed for intelligent fusion analysis of various indicators for in-school training items and several indices for career-required competence. The data has different presentations on a number of properties, such as variable type, data format, numerical difference, background knowledge, etc. [20]. These property inconsistencies will increase the difficulty of network learning. Confronting the nonuniform properties of different modules, the fusion analysis cannot be performed by simply listing them together, while some advanced fusion techniques are required [21]. The data belonging to each module has its own property, then a network weighted parameter is generated to adjust the input information of different modules. Then all input nodes are linked and transformed to the hidden layer. The number of hidden nodes is the key parameter of the network training structure. The network model can be adaptively optimized by testing a different number of hidden nodes. Simultaneously, the interactive layer linking weights are also for tuning during the network computation. In this way, the feature data extracted by the hidden neurons can have high-dimension identities with convenience in interpreting information [22, 23].

For quantification, the reference contribution matrix is acquired by discrete principal component analysis of the recorded scorings of the indices of career-required competence. The principal variables should be found for efficient analysis. Principal component analysis (PCA) is a frequently used method for extracting the main variable components [24]. However, most of the data records and the modeling indices are discrete, so the conventional PCA computing progress cannot deal with the discrete data [25]. Thus, a novel improvement is proposed for PCA to solve the multivariate modeling problem by observing the standard eigenvalues and eigenvectors in our study. A contribution matrix is defined as recording the scorings of the in-school training items contributing to the career-required job competence. This is regarded as the reference matrix for network modeling. On the other hand, the contribution matrix is predicted by the network training from the fusion of multiple modules of the in-school training items.

The aim of this work is to investigate the balance between the college's in-school training items and the career-required competence and successively evaluate whether the graduates have competent job abilities when they are employed by different companies at various posts. The data features are extracted to evaluate the difference between the predicted matrix and the reference contribution matrix. Further, the difference is taken as the indicator to evaluate whether the in-school training items are suitable to cultivate the high-quality talents that should have the competent career-required abilities. The modeling methodology provides theoretical guidelines for evaluating the fitness of the current cultivation mode performed on the college student.

The remainder of this article is organized as follows.  Section 2 describes the data source for college graduates' cultivation and sets up some relevant modeling indices.  Section 3 introduces the architecture of the adaptive neural network and the multitarget discrete PCA method.  Section 4 applies the adaptive multivariate neural network model to the data, for fusion evaluation of college cultivation.  Section 5 makes conclusions.

## 2. Data Preparation

### 2.1. Empirical Samples

A questionnaire was designed to collect sample data from recently graduated students of Guangzhou Colleges. The data involves four targets of employment postevaluation, i.e., Working location, Post, Salary, and Promotion times. These four terms are digitally transformed into ten terms for evaluating the career-required competence ability terms. On the other aspect, these ten terms are quantified with the fusion of the four data modules of at-school training items. Each career-required competence ability is quantitatively estimated with a seven-level rating. By normalization, each ability term could be scored as *i*/7, where *i*=1,  2,  3,  4,  5,  6,  7 represents Highest, High, Mid-High, Middle, Mid-Low, Low, and Lowest, respectively. Before model establishment and optimization, the data are for basic statistical analysis based on the partition, classification, or distribution of the four targets of employment postevaluation. We finally collected 1231 effective responses without any missing information.

Concerning the working location, the data show that most of the students selected to work in the 21 different cities in Guangdong province, and a few of them works outside Guangdong. We divided the 21 cities into 9 groups according to their Geographical location. Thus, we have statistical data for working location by 10 city groups (see Table 1).

For working posts, the data were classified into marketing, administration, technology, and management. There are 458 students (over one-third) working as technicians. Besides, there are 266, 284, and 233 students working in the marketing, administration, and management posts, respectively. They have nearly the same percentage of employment.

For salary payment, the 1231 employees were monthly paid ranging from 1,000 to 15,000 CNY. The full range is divided into 5 different levels of [1000, 3000), [3000, 5000), [5000, 7000), [7000, 9000), and [9000, +∞). Counts of employees distributed in these levels are 212, 697, 219, 67, and 36, respectively.

Promotion is another aspect to show whether the employees work hard and perform well. Of the 1231 samples, 70 students were promoted more than three times, 166 were promoted twice, 455 once, and 540 who paid less effort were never promoted.

### 2.2. Target Indices for Modelling

The graduates acquire the abilities through some in-school training items that are classified as data modules of courses, personal quality training, self-awareness development, and undergraduate experiences.  Table 2 shows that each module has different presentations in variable type, data format, numerical difference, background knowledge, etc.

To evaluate whether the graduate's ability supports their job competence, we designed a series of indices as the evaluation targets were made to accompany the fusion analysis of different data modules. The questionnaire questions highlight ten indices of career-required competence. They are (1) Teamwork, (2) Circumstance adaptation, (3) Communication, (4) Critical thinking, (5) Organization/Leadership, (6) Problem-solving ability, (7) Life-long learning, (8) Information search and processing, (9) Instant learning, (10) Innovation/Creativity. Each index was designed with seven-level scorings (i.e., Highest, High, Mid-High, Middle, Mid-Low, Low, Lowest). The respondents are required to tick a level of scoring would these indices support their current working posts. Simultaneously, the respondents should tick whether they have acquired these abilities from each item of their in-school studies. Therefore, these ten indices of career-required competence make the linkage between the job competency and the in-school items.

Thus, we built up the adaptive neural network to launch the fusion analysis of different modules for college student in-school cultivation on targeting the ten indices of career-required competence. Specially, we utilized the multitarget discrete PCA method to pretreat the data as most responses from the questionnaires are discrete records. Thus the models and the architecture established for fusion analysis should highly fit the data properties of different modules.

## 3. Methodologies

### 3.1. The Multitarget Discrete PCA Method

The typical PCA relies on the second moment, which is essentially similar to relying on the same mean value and the same variance. The direct introduction of discrete variables into PCA does not limit the computational range. Then the process no longer follows the assumption of normal distribution [26]. In this case, the Filmer-Pritchett method [27] is applied to find a single factor weighing the dependent variable.

For multitarget component analysis of discrete data with multiple distributions, we suppose the proportion of data in the *i*-th class is *τ*_*i*_ (*i*=1,2 … *n*), then the covariance matrix (**CovM**) of the independent variables is defined as follows:

(1) $$\begin{array}{c} CovM=\left[\begin{array}{c} \begin{array}{c} \tau_{1}\left(1-\tau_{1}\right)\\ -\tau_{2}\tau_{1} \end{array}\\ \begin{array}{c} \vdots \\ -\tau_{n}\tau_{1} \end{array} \end{array}\begin{array}{c} \begin{array}{c} \;-\tau_{1}\tau_{2}\\ \;\tau_{2}\left(1-\tau_{2}\right) \end{array}\\ \begin{array}{c} \vdots \\ \;-\tau_{n}\tau_{2} \end{array} \end{array}\begin{array}{c} \begin{array}{c} \;\cdots \\ \;\cdots \end{array}\\ \begin{array}{c} \;\ddots \\ \;\cdots \end{array} \end{array}\begin{array}{c} \begin{array}{c} -\tau_{1}\tau_{n}\\ -\tau_{2}\tau_{n} \end{array}\\ \begin{array}{c} \vdots \\ \;\tau_{n}\left(1-\tau_{n}\right) \end{array} \end{array}\right]. \end{array}$$

To simplify the computational process, we assume that *τ*_1_ > *τ*_2_ > …>*τ*_*n*_, then the covariance matrix can be transformed to the following:

(2) $$\begin{array}{c} CovM=\left[\begin{array}{c} \begin{array}{c} 1\\ -\mu_{21} \end{array}\\ \begin{array}{c} \vdots \\ -\mu_{n1} \end{array} \end{array}\begin{array}{c} \begin{array}{c} \;-\mu_{12}\\ \;1 \end{array}\\ \begin{array}{c} \vdots \\ \;-\mu_{n2} \end{array} \end{array}\begin{array}{c} \begin{array}{c} \;\cdots \\ \;\cdots \end{array}\\ \begin{array}{c} \;\ddots \\ \;\cdots \end{array} \end{array}\begin{array}{c} \begin{array}{c} \;-\mu_{1n}\\ \;-\mu_{2n} \end{array}\\ \begin{array}{c} \vdots \\ 1 \end{array} \end{array}\right], \end{array}$$

where $\mu_{ij}=\tau_{i}\tau_{j}/\sqrt{\tau_{i}\left(1-\tau_{i}\right)}\sqrt{\tau_{j}\left(1-\tau_{j}\right)}=\sqrt{\tau_{i}\tau_{j}/\left(1-\tau_{i}\right)\left(1-\tau_{j}\right)}$. Successively, the eigenvalues and eigenvectors of the discrete PCA procedure are obtained by solving the problem of *μ*_*ij*_.

Aiming to evaluate the job competency of the graduates, the discrete PCA methodology is used to weight the indices of career-required competence, respectively, based on the four factors for employment postevaluation (i.e., the working location, the post, the salary, and the promotion times). The covariance matrix of the independent variables is calculated for extracting the principal components, thus obtaining four covariance matrices (denoted as **CovM**(*fac*)_*n*×*n*_), where *fac* represents the different factors of the working location, the post, the salary, and the promotion times.

Then a scoring matrix is constructed to mark the 7-level scorings for each of the *n* classes (denoted as **ScorM**(*fac*)_7×*n*_). Also, a weighting matrix (denoted as **PW**(*fac*)_*n*×10_) is formed to digitalize the comprehensive scoring by proportion ratio of the 7-level for each class based on the 10 indices of career-required competence. Namely, the scoring contribution of the four covariance matrices to the evaluation of the 10 career-required competence can be demonstrated in the matrix multiplier as follows:

(3) $$\begin{array}{c} SM{\left(fac\right)}_{7\times 10}=ScorM{\left(fac\right)}_{7\times n}\times CovM{\left(fac\right)}_{n\times n}\times PW{\left(fac\right)}_{n\times 10},\\ \text{for }fac\in \left\{\text{working location,post},\text{salary},\text{promotion times}\right\}. \end{array}$$

For the convenience of network model training, we should create a novel covariance matrix with comprehensively weighting the importance of the four factors for employment postevaluation. According to the theory of information gain rate [28], the variable importance (VI) is proposed to quantify the importance weights of the four factors, which is defined as follows:

(4) $$\begin{array}{c} \text{VI}\left(fac\right)=\underset{k}{\sum }\tau_{k}\cdot \left(-\text{ln}\tau_{k}\right), \end{array}$$

where *k* represents the *k* th category under a certain factor, and *τ*_*k*_ represents the proportion of data in the *k*-th class (*k*=1,2 … *n*). Consequently, the comprehensive matrix (**CM**_VI_) for weighting the career-required competence can be identified as follows:

(5) $$\begin{array}{c} CM_{\text{VI}}=\sum_{fac}\text{VI}\left(fac\right)\cdot SM\left(fac\right), \end{array}$$

for each value of *fac* limited in a similar working location, a similar post, a similar range of salary, or a similar promotion times, respectively. Hereafter, the comprehensive matrix **CM**_VI_ is regarded as the contribution of the four factors for employment postevaluation to the ten indices of career-required competence. It enables the neural network model training performing for the prediction of the importance of in-school training items on the job competence.

### 3.2. The Adaptive Neural Network Architecture

The neural network is constructed in a fully connected structure (see Figure 1) for the full fusion of data information from different modules. An easy measure to integrate them is to design a weighted coefficient (*ρ*_*r*_) to render the ratio of the importance of different modules, where the subscript *r* screens the four data modules of courses, personal quality training, self-awareness development, and undergraduate experiences (i.e., *r*=1,  2,  3and4). Then the data of different modules are summed together with the weighted coefficients for network training. Each module contains a number of variables. Accordingly, the network fusion computations are modified.

All of the four modules are simultaneously delivered to the network input layer. There are a total of 32 variables describing the in-school training items. Each variable is normalized and taken as a single neuron node (denoted as *x*_1_, *x*_2_ … *x*_32_). With the summation calculation, the data delivered to the hidden layer is generated by the total summation of the fused input data. It can be formulated as follows:

(6) $$\begin{array}{c} {\text{net}}_{j}=\sum_{r=1,2,3,4}\rho_{r}\left(\sum_{x_{i}\in {\text{Module}}_{r}}w_{ij}\cdot x_{i}\right)+\theta_{j},\;i=1,2\ldots 32, \end{array}$$

where net_*j*_ is simply the summation and *w*_*ij*_ represents the weight evaluating the contribution of the 32 input variables to each of the feature variables at the *j*-th hidden nodes (denoted as *H*_*j*_, *j*=1,2 … *N*). Successively, the feature data is activated with the Sigmoid function [29], i.e.,

(7) $$\begin{array}{c} H_{j}=\text{Sigmoid}\left(net_{j}\right),\;j=1,2\ldots N. \end{array}$$

Moreover, the activated data of {*H*_*j*_}_*N*_ at the hidden neurons are further delivered into a Softmax unit. In the Softmax, the ten indices of career-required competence are evaluated by the *N* feature variables from the hidden layer,

(8) $$\begin{array}{c} i\;dx_{t}=\sum_{j=1}^{N}v_{jt}H_{j}+\sigma_{t},\;t=1,2\ldots 10, \end{array}$$

where *i*  *dx*_*t*_ is the *t*-th index and *v*_*jt*_ represents the linking weights of the hidden nodes and the ten indices.

Consequently, the softmax unit use Mahalanobis distance [30] to transform the information of the network-extracted feature variables to the targeting 7-level scoring values, thus observing the predictive value of the contribution matrix (**CM**_net_) for the implicit evaluation of the 32 in-school training items to the job competence of the graduates.

The network architecture is designed for adaptive optimization as the number of hidden nodes (*N*) is tunable. We could test some possible number of hidden nodes, compare the output results and find the most adaptive number. Practically, a good output result is identified when the contribution matrix meets as closely as possible to the abovementioned comprehensive matrix with variable importance (**CM**_VI_). Therefore, the second norm of the difference matrix (**M**_diff_) is used for the comparison. Then, it is mathematically evaluated as follows:

(9) $$\begin{array}{c} {\left\|M_{\text{diff}}\right\|}_{2}=\sqrt{\lambda_{max}\left(M_{\text{diff}}^{\text{T}}M_{\text{diff}}\right)}, \end{array}$$

where **M**_diff_=**CM**_net_ − **CM**_VI_, and *λ*_*max*_(·) is to find the maximum eigenvalue of a matrix. Thus the network model can be trained and optimized in a self-adaptive way, aiming to find the minimum value of ‖**M**_diff_‖_2_.

The network architecture is functional to perform fusion analysis of the data for the career-required competence ability and the in-school training items. The adaptive learning mode is held by the neural network structure, automatically fitting the linkage weights between each two linked nodes. The comprehensive **SM** and **CM** matrices are taken as for the error evaluation of the inherent covariance of the collected data. These advantages help to establish solid network models for rapid quantitative fusion analysis of the career-required competence ability of the graduated students and their in-school training items before graduation.

## 4. Results and Discussion

As for launching the adaptive neural network architecture, the reference contribution matrix was computed by the discrete PCA modeling methodology. The four target factors of employment postevaluation were transformed to be quantified with the 10 career-required competence ability terms, using the discrete covariance rating principle, thus generating a contribution matrix by fusion analysis of the four factors and the 10 indices.

Firstly, we calculated the data proportion (*τ*) in any class respectively based on each of the four factors. For the factor of working location, the 1231 samples were divided into 10 city groups. During the 10 classes, the 1231 graduates mainly work in Gz (G1), Sz (G2), Fs (G3), DH (G4), and OGD (G10). For the factor of working post, there concern four types of working posts (i.e., marketing, administration, technology, and management) in this study. The most employment is in the technology post. For the factor of salary, the data was presented as the normal distribution. The salary range that most of the 1231 graduates earn was [3000, 5000) when ignoring the influence of the other factors. For the factor of promotion times, we observed the phenomenon that there are over 70% of the graduates never promoted and only promoted once; only a few people promoted three times or more.

According to the theory and algorithm of discrete PCA, we have observed the value of *τ* for any of any divided class based on different factors of employment post evaluation (see Table 3). The values of *τ* were further used to calculate the covariance matrix and the scoring matrix of each class, and then the scoring contribution of the four covariance matrices to the evaluation of the 10 indices of career-required competence (**SM**) was computed using formula (3). The resulting **SM** values for each factor are shown in Figure 2, in which the value is evaluated by the rainbow color scale. We can visually acquire from Figure 2 the exact scorings for each index of career-required competence. Most graduates scored 4 or 5 for each of the factors of employment postevaluation. With interactive comparison, the scorings on working location were relatively higher than the other factors.

Next, the value of VI was calculated obeying formula (4) for each factor for employment postevaluation the VI's of each factor were estimated as shown in Figure 3. The VI for the working location is larger than the other factors, while the others are close to each other. This result demonstrates that the graduates just out of school are concerned much about the working location and relatively less about the other factors. Successively, the comprehensive contribution matrix **CM** was further computed based on the acquired **SM** matrices using the formula (5). With the weighting of VI, the matrix **CM**_VI_ represents the fusion modeling of the 7-level scorings on the 10 indices of career-required competence to interpret the combined computation effect of all of the four target factors. It is regarded as the job competence ability required by society based on the study of a fusion metric of the four different factors of employment postevaluation.  Figure 4 shows the scatter distribution of the computed **CM**_VI_ matrix values on the cubic axes of 7-level scoring and the indices of career-required competence. The matrix **CM**_VI_ was taken as the reference matrix for the following adaptive network training.

The constructed adaptive multivariate neural network structure was used for fusion analysis of data information extracted from the questionnaire-recorded 7-level scorings on 32 in-school training items. The 32 items were categorized in for different models. According to the adaptive training of the network architecture, the collected data for the in-school training items was renewed using the weighted coefficients of *ρ*_1_, *ρ*_2_, *ρ*_3_ and *ρ*_4_, respectively, for the four different modules of courses, personal quality training, self-awareness and undergraduate experience. Then, the renewed items were input to the neural network. The neural computation is to transform the input data into the hidden nodes, where the number of hidden nodes is for adaptive tuning. Considering that fewer hidden node is not sufficient to accept the feature information of data, we test the neural models with *N* changing from 5 to 20 in the hidden layer. Aiming to acquire the minimum different matrix (**M**_diff_) between the network predicted **CM**_net_ and the reference **CM**_VI_, the possible results of ‖**M**_diff_‖_2_ is showed in Figure 5 for the tuning of *N*. It is observed from Figure 5 that the optimal *N* equals 16, which indicates that the neural network constructed with 16 hidden nodes would have the best prediction results for evaluating the in-school training items contributing to the career-required competence. Simultaneously, the scatter values of the minimum **M**_diff_ is illustrated in Figure 6 projected to the 7-level scoring and the 10 indices of career-required competence based on the adaptive optimal network training model.  Figure 7 shows the distribution of the differences between the predictive **CM**_net_ values and the **CM**_VI_ values projection on the 10 indices of career-required competence and on the 7-level scoring, respectively. Most of the differences are low, and the maximum difference is less than 0.3. It indicated that the network predicted comprehensive contribution matrix for weighting the career-required competence is close to the matrix generated by discrete PCA multivariate transforming. The result proved that the students' working ability acquired from in-school cultivation items suits their career requirement.

The prediction results indicate some signals for the reform of student cultivation in colleges and universities in China. The in-school training items should be designed in close relation to the job competence. The quantified 10 indices show us that the cultivation of high-quality talents needs not only to impart the in-course knowledge but to enhance the training quality of the other modules is also much important. For example, the training in compressive ability, insights, and collaboration may enhance the students' personal quality. Instructing the way of self-positioning, career planning, and continuous learning is in much demand for raising students' self-awareness. Additionally, it is another key point to encourage the students to join clubs to participate in research project and international exchange.

In the sustainable development of cultivation reforming, the evaluation of how the in-school cultivations support the graduates' career-required competence is going to be more and more critical because college education in the future will be highly connected to the dynamic speed changing of the career-required competence in the information society. Experimental results have shown that the methodology based on the adaptive network fusion analysis is feasible to evaluate the balance between the in-school cultivation items and the career-required competence.

## 5. Conclusions

To evaluate the cultivation systems in colleges and universities, we proposed an adaptive multivariate neural network architecture for fusion analysis of the correlation between the in-school training items and the career-required competence. Firstly, we proposed to improve the PCA algorithm for discrete analysis. A series of covariance matrices were computed based on the factors of working location, working post, salary, and promotion times. Classifiers and 7-level scoring metrics were designed to transform the collected data into comprehensive data features for recording the contribution of the 10 indices of career-required competence, there to compose the reference contribution matrix for adaptive network learning. Next, a fully connected network structure was constructed for predicting the contribution matrix from the data of 32 in-school training items categorized in four modules. For data input, the network received data of different modules with weighted coefficients, then the data was delivered to the hidden layer. With the network linking weight adaptively trained, the number of hidden nodes was designed as the key tuning parameter for model optimization. Further, the contribution matrix was predicted by the feature variables acquired from hidden nodes, using the Mahalanobis distance. Finally, the network-predicted contribution matrix was compared to the reference matrix, using the second norm of the difference matrix as the quantifier.

Experimental results show that the methodology of adaptive network fusion learning is feasible to provide a novel system for modeling evaluation of whether the in-school training items support the career-required competence of graduates. The fused feature extracted from different module data, the intelligent training of network linking weights, and the prediction of the norm of the difference matrix help to explore the implicit work competent abilities hidden behind the in-school training items. The proposed computing framework lays a good foundation for revealing the direct correlation of college cultivation and job-required abilities. We wish to let the undergraduate students study positively and initiatively, stimulate their interest and power in the study, and simultaneously give directions and positive suggestions for colleges and universities to make their cultivation reforming as to enhance the quality of their graduates.

In the future, we plan to further explore the relationship between the in-school training items and the career-required competence ability by comparing the correlation effects (including the coefficient of data, coefficient of variation, and coefficient of the PCs) along with the covariance matrix, to explore the more deep inherent relationship. Furthermore, we will investigate other modeling methods such as the swarm intelligence evolution algorithms and decision tree-entropy modification methods.

## Figures and Tables

**Figure 1:** The neural network structure for fully connected training.

**Figure 2:** The SM value predicted by discrete PCA model. (a) for working location (b) for working post (c) for salary (d) for promotion times.

**Figure 3:** The variable importance of the four employment post evaluation factors.

**Figure 4:** The **CM**_**VI**_ matrix calculated based on VI for comprehensive evaluation on the career-required competence indices.

**Figure 5:** The network predictive difference matrix by tuning the number of hidden nodes.

**Figure 6:** The prediction of **M**_diff_ based on the adaptive optimal network training model.

**Figure 7:** Differences between the **CM**_net_ and the **CM**_VI_ values projection on the 10 indices of career-required competence and on the 7-level scoring.

**Table 1:** City group partitioned by employment data.

City group (abbreviation)	Number of employment
Guangzhou (Gz)	370
Shenzhen (Sz)	197
Foshan (Fs)	117
Dongguan, Huizhou (DH)	126
Outside of Guangdong (OGD)	138
Jiangmen, Zhongshan, Zhuhai (JZZ)	77
Maoming, Yangjing, Zhanjiang (MYZ)	57
Qingyuan, Yunfu, Zhaoqing (QYZ)	38
Heyuan, Meizhou, Shaoguan (HMS)	46
Chaozhou, Jieyang, Shantou, Shanwei (CJSS)	65

**Table 2:** The in-school training items when undergraduate.

Module	Item
Courses	Professional technique
	General course
	Innovation and entrepreneurship
	Practical course
	Double degree program
	Academic guidance
	Career guidance
	Scientific research introduction

Personal quality training	Compressive ability
	Circumstance adaptation
	Insight
	Capability of information screening
	Strategic planning
	Sense of responsibility
	Loyalty
	Collaboration

Self-awareness	Self-positioning
	Career planning
	Job search
	Self-marketing
	Continuous learning
	Resource control

Undergraduate experience	Club activity
	Social practice
	Leadership experience
	Academic lecture
	Science competition
	Research project
	Cultural/sport activities
	Volunteer
	International exchange
	Award

**Table 3:** The values of *τ* of any divided class based on different factors of employment post evaluation.

Working location		Gz	Sz	Fs	DH	JZZ	MYZ	QYZ	HMS	CJSS	OGD
	*τ*	0.3006	0.1600	0.0950	0.1024	0.0626	0.0374	0.0463	0.0309	0.0528	0.1121

Working post		Marketing		Administration		Technology		Management		—	—
	*τ*	0.2161		0.2307		0.3721		0.1812		—	—

Salary		[1000, 3000)		[3000, 5000)		[5000, 7000)		[7000, 9000)		[9000, +∞)	
	*τ*	0.1722		0.5662		0.1779		0.0544		0.0292	

Promotion times		Never		Once		Twice		≥ Three times		—	—
	*τ*	0.4387		0.3696		0.1348		0.0569		—	—

## Data Availability

The data used to support the findings of this study are available from the corresponding author upon request.
